# General practitioner contributions to achieving sustained healthcare for offenders: a qualitative study

**DOI:** 10.1186/s12875-018-0708-7

**Published:** 2018-02-02

**Authors:** Cath Quinn, Katie Denman, Philippa Smithson, Christabel Owens, Rod Sheaff, John Campbell, Ian Porter, Jill Annison, Richard Byng

**Affiliations:** 1 Plymouth University, Drake Circus, Plymouth, Devon PL4 8AA UK; 2 University of Exeter Medical School, St Luke’s Campus, Exeter, EX1 2LU UK

**Keywords:** General practitioner, Primary care, Access, Continuity, Offenders, Qualitative

## Abstract

**Background:**

Offenders frequently have substantial healthcare needs and, like many other socially marginalised groups, often receive healthcare in inverse proportion to their needs. Improved continuity of healthcare over time could contribute to addressing these needs. General Practitioners need to be able to support people with complex social and medical problems, even in systems that are not specifically designed to manage individuals with such degrees of complexity. We aimed to examine offenders’ perspectives on factors that contributed to, or worked against, creating and sustaining their access to healthcare.

**Methods:**

From a sample of 200 participants serving community or prison sentences in South West (SW) and South East (SE) England, who were interviewed about their health care experiences as part of the *Care for Offenders: Continuity of Access* (COCOA) study, we purposively sampled 22 participants for this sub-study, based on service use. These interviews were transcribed verbatim. A thematic analytic approach initially applied 5 a priori codes based on access and different components of continuity. Data were then examined for factors that contributed to achieving and disrupting access and continuity.

**Results:**

Participants described how their own life situations and behaviours contributed to their problems in accessing healthcare and also identified barriers created by existing access arrangements. They also highlighted how some General Practitioners used their initiative and skills to ‘workaround’ the system, and build positive relationships with them; feeling listened to and building trust were particularly valued, as was clear communication. Limitations faced by General Practitioners included a lack of appropriate services to refer people to, where the offender patients would meet the access criteria, and disagreements regarding medication prescriptions.

**Conclusions:**

General Practitioners can make a positive contribution to supporting access to healthcare for an under-served population by facilitating more flexible and less formal access arrangements, by using their relationship skills, and by problem-solving. General Practitioners should recognise their potential to transform people’s experience of healthcare whilst working in imperfect systems, particularly with vulnerable and marginalised groups who have complex medical and social needs.

## Background

Offenders, like homeless populations, frequently have substantial health needs, particularly relating to mental health and substance misuse [1–5]. As with other socially marginalised groups, they often receive healthcare in inverse proportions to their needs [6–8]. The United Nations recommends that prisoners are given equitable access to healthcare (Principle 9, A/RES/45/111) [9]. In the United Kingdom, although the National Health Service (NHS) has overall responsibility for prison healthcare, physical health, mental health and substance misuse services are still usually commissioned and provided separately. Arrangements for transitions from prison to community care are often absent. In the community, care is provided by mainstream NHS services, usually by General Practitioners in primary care teams and by separate substance misuse services, with minimal access to specialist mental health services.

Offenders can be a challenging population to work with both emotionally and practically; they are likely to experience numerous social problems including homelessness and financial difficulties [10, 11]. Offenders have been shown to be reluctant to access healthcare due to previous negative experiences, which have contributed to their distrust of ‘the system’ and authority figures and, in the case of mental health services, a fear of stigmatisation [12]. Although those working in substance misuse services may be aware of an individual’s criminal justice involvement, General Practitioners are not routinely given this information and may be treating such patients, including those with experience of incarceration, without being aware that they are doing so.

Freeman et al., have defined continuity of healthcare as dependent on continuity of access and these 4 elements: 1) Relational continuity, both personal and therapeutic; 2) longitudinal continuity, the provision of healthcare over time; 3) flexible continuity, care adjusting to changes in a person’s life; and 4) continuity of communication including information and working relationships, and between professionals and across teams and statutory boundaries [13, 14]. Continuity of healthcare over time for socially excluded groups has received minimal research attention, despite their being one of the groups with the greatest potential to benefit from this, due to high levels of healthcare need and comparatively low levels of healthcare received.

This qualitative study explores the offender participants’ experiences of what does and doesn’t work in gaining initial and ongoing access to healthcare. We highlight how General Practitioners, working with imperfect systems and individuals with challenging and complex needs, can make a positive contribution to healthcare for offenders and we suggest how sustained access to healthcare might be improved for this under-served group.

## Methods

This paper reports a qualitative analysis of interviews with 22 offenders about their healthcare. We aimed to examine what, from the participants’ perspectives, contributed to, or worked against, achieving sustained access to healthcare for offenders. We conducted interviews, which included a mixture of open and closed questions, with 200 offenders in 2 contrasting English localities (SE & SW England) as part of the Care for Offenders: Continuity of Access (COCOA) study. The study report includes a copy of the interview schedule [6]. Interviews took approximately 1 h and were carried out by one male and three female researchers working on the wider COCOA project; 3 had PhDs (Doctor of Philosophy) and one had a Master’s degree, all had experience of conducting research with vulnerable groups and had received training in working with offender populations. The researchers did not know the participants prior to the interviews. We recruited participants at the start of community sentences (*n* = 100), and the start (*n* = 50) and end (*n* = 50) of prison sentences. Interviews were conducted in a private room and justice staff were not present. The participants were asked a mixture of open and closed questions about their social and economic situation, their contact with the Criminal Justice System (CJS), any illnesses, and their contact with healthcare services over the past 6 months. When feasible, follow-up interviews were carried out at approximately 3 and 6 months to record repeated measures of healthcare contact and any emergent health problems. Participants were interviewed face-to-face using a conversational style of delivery to facilitate participation. Interviews were digitally audio recorded, when possible. The closed questions produced data suitable for quantitative analysis [6]. The open questions and the general conversations about answering the closed questions produced rich accounts of the participants’ experiences which were suitable for deeper qualitative analysis. From the wider sample, we purposively selected a sub-set of participants who reported high levels of contact with: i) Physical health services; ii) mental health services; iii) substance misuse services; and iv) low levels of overall healthcare contact. Only male participants were selected for this sub-study because of the low numbers of women (*n* = 20) in the overall sample. Twenty-two participants were selected, of whom four had one follow-up interview. The audio recordings of these 26 interviews (22 + 4) were transcribed verbatim. The participants ranged in age from 19 to 59 years old. Ten had partners and 11 had children under the age of 18. Six were serving community sentences, nine were serving the start of a prison sentence and seven were due to be released from prison soon.

We applied an interpretive thematic approach to analysing these transcripts, starting with 5 a priori codes based on Freeman et al.’s four components of continuity (relational, longitudinal, flexible, communication) and access. We use the term ‘access’ to refer to both initial and continuing access throughout this article. Two qualitative researchers (CQ and KD), with some knowledge of the CJS, checked and confirmed each other’s coding to promote consistency and reliability; differences were resolved by further discussion. Nvivo8 software was used to group the relevant data. Working with 2 General Practitioner researchers with clinical experience of working with this group (PS and RB), we explored the participants’ reasons for, and experiences of, accessing healthcare; or choosing not to. Saturation in the analytical process was considered to have been reached when no new ideas emerged in the discussions between CQ, KD, PS and RB. We compared these findings with Freeman et al.’s original definitions and identified that the health and criminal justice systems, the offenders themselves, health practitioners (particularly General Practitioners) and some justice practitioners were the key components in promoting or disrupting access to healthcare for offenders. The contribution of each of these components is detailed in the results section, below.

## Results

Freeman et al.’s conceptualisations of the components of continuity, to achieve sustained access, are ideal types; they do not take into account the moderating influence of the interactions between imperfect systems and actors. Our analysis demonstrated the contributions of the following to promoting and disrupting access to healthcare for offenders:

i) The offenders’ contributions.
ii) The health and justice systems contributions: Access arrangements and communication.
iii) Individual General Practitioners: Mitigating difficulties and disruptions.
iv) Limitations faced by General Practitioners.

### The offenders’ contributions

Participants recounted their contributions to both promoting and disrupting their own access to healthcare. Promoting access included examples of participants’ persistence despite encountering organisational obstacles. One participant repeatedly contacted an alcohol service which had offered him an appointment and a key worker:

“I went down there and I was buzzing the bell and no one answered, so I went and rang them and no one answered the phone so I left a message and then rang back the next day and the next day” (2003a).

Accounts of disrupting their access to healthcare included a participant having their methadone (heroin substitution) prescription withdrawn, after repeated warnings, due to excessive use of alcohol (1027a). Other participants had rejected the healthcare they were receiving because they did not like the manner in which it was delivered; their accounts implied that they felt scared and unable to cope with the situation. One participant didn’t want a camera put down his throat for a suspected ulcer without being sedated, so he walked away from the hospital (2003a). Some participants described how they were dissuaded by obstacles that others might perceive as a minor inconvenience, “I did go to see my doctor and ask for an appointment for tablets to stop my drinking … but I was told to come back in a week’s time so I didn’t bother” (1015a), and “If you get a hospital that’s miles away and you’ve got to get to them you’ve got to say you’d rather not go” (2048a). Other participants no longer sought support from the health system because of previous bad experiences, “If I, if I get any problems I just won’t bother seeing them because, that’s just the way I feel. They’ve never done anything really for me in the past, not really” (1117b).

### The health and justice systems contributions: access arrangements and communication

Access for seemingly straightforward problems can be complex for some individuals. Participants reported using direct-access services such as ambulances and Accident and Emergency departments, for conditions that could have been cared for in primary care. A participant in his 20s described going to a hospital when he needed an inhaler for his asthma “because I’d run out, so I went down the hospital and said ‘Can, can I just have an inhaler?’ I said ‘That’s all I need’” (2003a). Another participant in his 20s telephoned for an ambulance because he thought he was having a heart attack; this request was refused so he walked to the hospital where he was told he had an irregular heartbeat and should see his General Practitioner. He expressed frustration that healthcare was not there for him when, and in the form, he felt it should be (1146a). Participants reported difficulties navigating the healthcare system; one participant expressed a desire for a key-worker who would remove the need for him to “get in touch with so and so… getting this from there or that from there”, which he found difficult (1036a).

Participants experienced difficulties in sustaining access to healthcare when they moved between different services for the treatment of the same problem; these challenges were exacerbated by the participants’ life situations. A participant in his 40s, who had been warned that he would be dead within a year if he did not stop drinking, had tried to access support but was frustrated that this resulted in being placed on waiting lists, “oh well I’ll wait but while I am waiting I’ll keep drinking” (1004a). Moving in and out of prison also disrupted some participants’ continuing access to healthcare. Entering prison led to interruptions or changes in medication, particularly if a prisoner arrived outside of office hours, which caused delays in receiving information from community health services. Imprisonment also disrupted on going relationships with community based health practitioners and previous referrals to community services. Some participants used incarceration as an opportunity to purposively address their health needs, including detoxification, vaccination, weight gain and breaks from heroin use, “sometimes I ask to go to jail just to sort me head out and get clean” (1027a). Healthcare was described as being easier to access in prison, due to higher staffing levels, and care being available 24 h a day. Subsequent release from prison, however, disrupted ongoing access to healthcare, particularly if there were no arrangements for the support provided in prison to be maintained in the community.

“I did detox, come out, there wasn’t any help afterwards so I relapsed and got back on it … it happens all the time ‘cos I’ve seen it happen to so many people before. They’ve come out and they’re clean and then they haven’t got anywhere to live, they’re on the streets and the next thing you know they’re back on the drugs again” (2029a).

Communication with health services can be difficult for the general population; offenders’ frequently challenging life situations can make this communication even more problematic. Participants who had been homeless reported failing to receive appointments and struggling to register with a General Practitioner.

“I haven’t received the actual appointments themselves … they have sent them out but I haven’t got them … because I have been like staying in different places … I did have an appointment to see a psychiatric nurse a week before I got sent down, but I missed the appointment because I was homeless at the time” (1015a).

Several participants mentioned poor communication between health services, particularly between prison and community prescribers, as impeding ongoing access to healthcare. Communication from services to offenders was emphasised as being particularly important to participants, “I asked [*name of prison doctor*] and she was going to contact my doctor on the out [*outside prison*], and I give her the number and that, but I haven’t heard nothing back off her” (1135a).

### Individual general practitioners: Mitigating difficulties and disruptions

Participants’ positive descriptions of healthcare generally included an account of a General Practitioner’s initiative, in either changing the ways in which services were delivered or in how they applied their medical skills. More flexible and less formal access arrangements had been achieved by local arrangements which located primary care services in places that offenders were already attending, such as CJS settings or homeless shelters. One participant described how he had only accessed healthcare because *“*there’s a doctor that comes to the hostel”; he had not tried registering with any other doctor (1135a). Co-location of services, for example an alcohol support nurse attending a probation service office, meant that the man who would otherwise have been deterred by waiting lists (above), eventually received help in addressing his alcohol dependency “I used to have to go to (*name of SW hospital*) that’s miles away, so but people have helped me, like you say the nurse can come here … so to come here is, you know, easier” (1004a).

Offender participants reported appreciating feeling listened to, and understood, by General Practitioners who spent time with them; they also valued what could be described as good all round medical care, such as receiving treatment, referrals and information. One man explained that, on being accused of rape, he valued his doctor’s supportive and practical approach, “the advice that he give me and knowing that he said if I ever need him, I can just go up there and speak to him” (2003a) left him feeling that he could go to his doctor if he had further problems. General Practitioners showing initiative and acting on behalf of, and in the interests of, participants were also experienced as demonstrating care (1117b). General Practitioners promoting a sense of trust were described as being important in participants’ willingness to use healthcare services. Straightforward, clear communication by General Practitioners was also valued: both directly with the offender, and when General Practitioners kept them up to date about their wider healthcare such as referrals (1099a).

Accounts of proactive practitioners working around the system to support offenders included Criminal Justice staff. “I got on well with the officers anyway, and one of them had gone off duty and she phoned the prison ... and said has he had any tablets and they said no, she went mad, cos she’s gone home but she knew what the system was like and what had happened” (2048a). Criminal Justice practitioners helped offenders to negotiate healthcare systems that the organisation of those systems, or their own predispositions, might have obstructed them from. “She [*Probation officer*] got in touch and then automatically I got the appointment” (1178a).

### Limitations faced by general practitioners

Limitations faced by individual General Practitioners included their being unable to access services for offender participants when an appropriate service, for which the participant met the access criteria, did not exist and when there were differences in opinion between the participants and their General Practitioners. These disagreements often focused on medication; one participant recounted:

“Because she was saying to me if you don’t stop the drugs you are taking at the moment I will stop your script and I said well if you stop my script then you are going to make me turn back to crime to feed my habit to take drugs” (1014a.)

These disagreements did not, necessarily, focus on a lack of care but on the participant rejecting the General Practitioners’ emphasis on following opiate substitution prescribing guidance, and their concern to promote wellbeing through engaging in less harmful behaviours (1036a). Prescribing can be a particular point of tension for practitioners working with individuals with complex needs, requiring skilful, assertive, person-centred and caring negotiation.

## Discussion

We have explored how offenders, practitioners (particularly General Practitioners) and the health and justice systems have contributed to maintaining and disrupting initial and ongoing access to healthcare for offenders. The key findings detail how General Practitioners have, in the absence of a single effective and connected system, managed to make a difference by facilitating more flexible and less formal access arrangements, by using relationship skills (demonstrating listening and understanding, spending time and building trust) and problem-solving (acting on behalf of and in the interests of offenders, communicating with offenders and other services and negotiating healthcare systems) [15]. Individual initiative alone, however, cannot achieve sustained access to healthcare for offenders more widely and systematically. Individual initiative and skills were also not always able to overcome differences in opinion between offenders and practitioners as to what constitutes good medical care, particularly in relation to the prescribing of medication. We focused on the perspective of offenders, which is a strength, in that it highlights a marginalised social group’s experience, but also a limitation, in that this article only considers offenders’ perceptions. The results report only the contributions of 22 purposively selected male participants. Offenders who did not speak English, were female, or below 18 years old, were excluded from this study.

Recent research [16–18] and our initial coding have emphasised flexible and relational continuity as key facets of continuity. We demonstrated that practitioner flexibility and relationship skills, along with flexible organisational arrangements, can also be seen as contributors to initial and ongoing access to care and treatment. Our study corroborated other researchers’ findings of the importance of both offender and organisational contributions to healthcare access [19–21]. Positive relationships have been shown to contribute to the continuity of care of vulnerable patients [22], we went further by highlighting how practitioners can potentially overcome offenders’ contributions to discontinuity. We demonstrated that strong personal relationships were experienced as contributing to good care and corroborated the assertion that trust and feeling listened to are particularly important to male offenders [12]. Our findings also support earlier research [21], showing the presence and nature of organisational obstacles to continuity of care for offenders. Vulnerable populations accessing primary care in the United States also identified poor information flow and misalignment of goals, between healthcare staff and patients, as contributing to a poor experience of care [23]. We noted that offenders described clinicians enacting ‘workarounds’ to overcome organisational barriers [24, 25].

## Conclusions

This research provides further evidence about the crucial importance of General Practitioners building trust and understanding with offenders and other socially marginalised groups, who are likely to receive comparatively low levels of healthcare for their substantive healthcare needs. These ‘inverse care’ groups have, potentially, the most to gain from improved and sustained access to healthcare. General Practitioners may be unaware of which of their patients have experience of justice involvement or incarceration and should consider working in this way with all patients whose complex social needs interact with their medical needs. General Practitioners need to be aware that their behaviour can influence individuals’ access to healthcare and to recognise that flexibility, clear communication and demonstrating empathy, as well as being good practice, also help address the specific problems faced by offenders, and other vulnerable or marginalised populations, in obtaining healthcare. Healthcare managers and practitioners working with these groups might consider ways in which they could be more flexible in their appointment systems and with arranging referrals. Having seen what is being achieved, we need a better understanding of what is beneficial to enact with imperfect systems and vulnerable populations, and where we should be concentrating our efforts to improve access arrangements. Further research should be undertaken into the organisational conditions producing the disruptions to continuity of care and potential remedies for health service systems should be identified. These findings could then be used to inform both health and justice policy.

## Abbreviations

CJS: Criminal Justice System
COCOA: Care for Offenders Continuity of Access
NHS: National Health Service
PCT: Primary Care Trust
PhD: Doctor of Philosophy
SE: South East
SW: South West
